# Application of Graphic Design with Computer Graphics and Image Processing: Taking Packaging Design of Agricultural Products as an Example

**DOI:** 10.1155/2022/6554371

**Published:** 2022-06-02

**Authors:** Tianhe Xie, Rongyi Sun, Jiahao Zhang, Ruiqi Wang, Jiashu Wang

**Affiliations:** College of Landscape Architecture and Art, Northwest A&F University, Xianyang 712100, China

## Abstract

With development of economy, all industries have undergone earthshaking changes. Various new technologies are starting to be employed in all aspects of life, and graphic design is no exception. The use of computer graphics and image processing technologies in graphic design can substantially improve design efficiency and make graphic design job more convenient to develop. The requirements for the quality of graphic design are higher. Quality inspection has become a necessary step in the production process, in which the detection of graphic design defects is an indispensable and important link. The traditional graphic design defect detection adopts the method of manual visual inspection, which has the disadvantages of poor stability, long consumption time, and high labor cost. As an efficient computer graphics and image processing technology, convolutional neural network has received extensive attention in graphic design defect detection because of its advantages of high speed, efficiency, and high degree of automation. Taking agricultural product packaging as an example, this paper studies application technology for graphic design defect detection with convolutional neural network (CNN). The main contents are as follows: construct the original YOLOv3 network model, input the graphic design images of agricultural product packaging into the network model in batches according to the computing power of the hardware equipment, train the YOLOv3 network, and deeply study and analyze the experimental results. The related improvement techniques are then given, based on the characteristics of agricultural product packaging design faults. The backbone network, multiscale feature map, a priori frame, and activation function of YOLOv3 are improved, and then performance of the improved model is verified by experiments.

## 1. Introduction

At this point, the development and applicability of computer graphics and image processing have made graphic design work much easier. Computer graphics and image processing technology have rapidly become an essential competence for designers in the work process in the graphic design business. Various picture information may be modified and optimized in terms of style, color, and theme using this technology, which can not only enhance the design effect but also improve job efficiency, effectively encouraging the design industry's development. The application of computer graphics and image processing technology in graphic design can solve the problems of diversity and aesthetics in graphic design to a certain extent and can also add more richness to the content of graphic design. In the process of using computer graphics and image processing technology, it is necessary to fully exploit the role and value of computers. However, we must also realize that there are still many unreasonable problems, which cannot give full play to the role of computer graphics and image processing technology, which affects the sustainable and healthy development of graphic design. Among them, graphic design defects have become a long-standing problem, and most graphic design products have certain defects. How to detect the defects of graphic design products has become an important and practical topic [1–5].

Manual quality inspection is still widely used, especially in small and medium-sized businesses that use human detection methods, and it accounts for a significant portion of the market. Manual quality inspection, on the other hand, must remain in a fixed position, which can lead to a variety of inspection issues when determining the presence of flaws by eye observation. Manual quality inspection cannot even ensure the stability and consistency of the detection of the same batch of graphic design products due to the influence of factors such as individual variances. In addition, missed detection and false detection are prone to occur during the detection process, the accuracy of the detection results is reduced, and the product quality is uneven. In addition, the upper limit of manual inspection efficiency is low, the cost is high, and a sampling inspection strategy is usually adopted to ensure production efficiency. The quality assessment of the entire product group by randomly selecting several products from the same group of products is far less rigorous than large-scale testing. Therefore, in the manual quality inspection process, quality control and production efficiency cannot always be achieved at the same time. In addition, defect detection requires not only qualitative inspection of the appearance of graphic design products but also statistics of defect size and other data. However, manual quality inspection can only rely on paper and pen to record, and the obtained data is not comprehensive and cannot be used as valuable information to guide production and production optimization and improvement [6–10].

Machine vision detection technology is a modern detection technology that integrates photoelectric sensing, computer science, image processing, pattern recognition, and other disciplines. It converts the captured target into an image signal, transmits it to a dedicated image processing system, and extracts the parameters to be detected, thereby realizing the defect detection of graphic design products. Machine vision inspection technology offers many advantages over hand visual inspection: noncontact measurement of the product to be inspected causes no damage to the product. The wider spectral response range and higher resolution extend the visual range and resolution of the naked eye. Stable, reliable, and fast work for a long time makes up for the shortcomings of poor visual stability and low work efficiency. The mechanized nature has greatly increased the degree of industrial automation. In recent years, due to the rapid development of machine vision and digital image processing, defect detection technology based on machine vision has received more and more attention in industrial quality inspection and has been widely used in various industries. Based on the above background, it is of great significance to study the defect detection technology of graphic design based on machine vision [11–15].

This work offers a computer graphics and image processing technology based on convolutional neural networks to detect faults in agricultural product packaging design, using the packaging design of agricultural products as an example. The characteristics of surface defects in agricultural product packaging design are studied in depth in this research, and then enhancements to the network model, feature maps, prior boxes, and activation functions are proposed. Finally, the revised network model is experimentally tested and compared to the original network model's experimental results. The results show that the improved network model can improve the detection accuracy of agricultural product graphic design defects.

The paper's organization paragraph is as follows: the related work is presented in Section 2.  Section 3 analyzes the methods of the proposed work.  Section 4 discusses the experiments and results. Finally, in Section 5, the research work is concluded.

## 2. Related Work

Reference [16] proposed a real-time algorithm for weaving defect detection based on machine vision. The technique detects five types of fabric surface defects using image processing methods such as wavelet transform, double-threshold binarization, and morphological operations, with a 93.4 percent defect detection and 96.3 percent defect type identification accuracy. Reference [17] proposed a camshaft surface defect detection method based on neighborhood weighted segmentation. The method realizes the detection of typical defects such as trauma, trachoma, and poor grinding on the surface of the camshaft through defect segmentation and defect area marking. At a speed of 0.44 s per shaft, the method was able to detect defects larger than 1 mm in diameter on the camshaft surface. Reference [18] proposed a method for detection of bottle mouth defects based on threshold segmentation, which combines three-circle positioning method, residual analysis dynamic threshold, and global threshold segmentation to detect five kinds of bottle mouth defects. Reference [19] adopts NCC for defect detection and adopts the integral graph strategy to speed up the traditional NCC calculation, so that the calculation time does not change with the change of the template window size. Reference [20] proposed an engine block defect detection based on small area template matching. The method combines rough search and fine search strategy improvement algorithm to determine the exact position and similarity of the images to be matched, realizes defect detection, and has a faster operation speed and meets real-time requirements. Reference [21] proposed a method for detecting appearance defects of smart meters based on machine vision. The method uses image processing technologies such as median filtering, binarization, edge detection, template matching, and OCR to detect the defects of smart meter LCD screen, signage characters, barcodes, and LED indicators, and the detection takes 3 s. Reference [22] proposed a keyboard defect detection method based on template matching. The method utilizes local threshold segmentation and coordinate projection to locate keys and uses template matching to match key characters to realize keyboard defect detection. Reference [23] proposes a steel surface defect detection algorithm, which uses Hough transform, PCA, and self-organization map to detect three kinds of steel surface defects, and achieves an 87% accuracy on the Arcelor Mittal image set. Reference [24] proposed a TFT-LCD defect detection algorithm based on machine vision. The algorithm uses Gabor filtering, adaptive binarization, connected domain extraction, and blob algorithm to identify TFT-LCD point defects and line defects and achieves a high recognition rate. Reference [25] proposed a fabric defect detection method based on SVM. The method extracts the geometric features of the fabric surface pattern and uses the SVM classifier to achieve defect detection, which can detect 5 kinds of fabric defects with an accuracy of 94.84%. Reference [26] proposed a defect detection and identification algorithm based on the PCA algorithm, which was applied to the surface of unshaded cover glass. Algorithms combine surface defect detection and identification processes into one. The missed detection rate and false alarm rate in the defect detection process reached 12% and 6%, and the recognition rate in the defect identification process reached more than 90%. Reference [27] proposed a defect detection algorithm based on CNN variant network Overfeat.

The algorithm uses Overfeat CNN combined with ASR for surface defect detection and achieves 98.7% and 60.3% accuracy on NEU and MO databases, respectively. Literature [28] developed a welding seam detection method based on multilayer perceptron and achieved good detection results on its data set. Literature [29] studied a variety of surface defect detection techniques based on texture feature extraction and summarized the progress of anomaly detection methods in the field of texture detection. Reference [30] used fractal dimension as feature quantity in hot-rolled strip surface defect identification and estimated an optimal scale to detect defects through fractal dimension curve graph to obtain better detection effect. Reference [31] proposes a method for detecting foreign matter in liquid medicine based on the idea of difference between frames, which achieves high detection accuracy and speed. Convolutional neural networks based on deep learning have demonstrated their powerful capabilities in feature extraction and pattern recognition; so, more and more defect detection methods incorporating deep learning have emerged. Reference [32] developed a visual inspection device for inspecting cigar pack labels at a speed of 500 packs per minute. Reference [33] used texture analysis to detect the seal quality of food packaging bags.

## 3. Method

This work uses convolutional neural network as a computer graphics image processing technology to detect the defects in the graphic design of agricultural product packaging. The convolutional network used is YOLOv3, and a series of improvement measures have been taken to effectively improve its performance.

### 3.1. Convolutional Neural Network

CNN is an artificial neural network designed to imitate the working mode of neurons in the human brain. The basic unit is artificial neurons. Artificial neurons also transmit signals hierarchically and perform extremely well when dealing with gridded data, especially for large image processing. Convolutional neural networks usually include the following structures: input layer, convolutional layer, pooling layer, fully connected layer, and output layer. The input layer is responsible for the input of the network, which is generally a matrix of numbers representing an image. The image input to the network will then go through a series of convolutional layers, pooling layers, and fully connected layers, and finally, the output layer will input the result.

The convolutional layer is an important part of the convolutional neural network, and the layers are directly connected locally to map the underlying information into high-level features. Each convolutional layer has multiple convolution kernels, and the size and number of convolution kernels have an important impact on the recognition ability of the convolutional neural network. The essence of a convolution kernel is a set of trainable weight matrices. When convolution operation is performed on the input image, the convolution kernel covers part of the input image according to a certain rule, and the value of the convolution kernel is multiplied by the value of the corresponding position pixel in the image. Adding the products obtained in the previous step is the result of this convolution operation. Convolutional layers are often used to extract image features, and the result after a series of convolution operations is often referred to as a feature map. The mathematical expression of the convolution operation is as follows:

(1) $$\begin{array}{c} y_{j}^{l}=\sigma \left(\sum x_{i}^{l-1}*w_{ij}^{l}+b_{j}^{l}\right). \end{array}$$

Weight sharing is an important feature of the convolution layer. Weight sharing means that when performing convolution operations, all positions of the image use convolution kernels with the same parameters. Weight sharing drastically decreases the network's parameters, allowing for much faster model training and inference. Another element of the convolution layer is multiconvolution operation, which refers to the employment of multiple separate convolution kernels to scan the input image. The scan result of each convolution kernel is a feature map, and finally, the multifeature map is used for prediction, and the accuracy can be greatly improved.

The pooling layer is generally located after the convolutional layer, and its main function is to compress the size of the feature map to reduce the amount of network parameters. The output of the pooling layer is the same as the convolutional layer, which is a feature map. These feature maps uniquely correspond to a feature map of the previous layer, and the size will be reduced to a certain extent. In theory, it is possible to directly input the feature map output by the convolutional layer into the classifier for result prediction. However, after the convolution operation of the image, the size of the image is not significantly reduced. Instead, due to the convolution operation of multiple convolution kernels, the feature map of the network increases. This increases the number of network parameters and the amount of computation, which seriously affects the training speed of the network. Therefore, it is necessary to perform a dimensionality reduction operation on the convolutional feature map, which is called a pooling operation. Pooling is the use of filters to filter out invalid information in the feature map after convolution operation, saving important information while reducing the amount of information and complexity. The pooling operation has strong advantages in reducing network parameters, reducing the amount of computation, and enhancing the robustness of the network. The pooling operation is as follows:

(2) $$\begin{array}{c} y_{j}^{l}=\text{down}\left(y_{j}^{l-1}\right). \end{array}$$

The pooling operation first divides the feature map into small matrices of equal size and does not overlap and then selects a value to replace the entire small matrix according to different criteria. There are two commonly used criteria, one is max pooling, which is to keep the one with the largest element in each small matrix. The second is average pooling, which is to average and retain all elements in each small matrix. After the feature map is pooled, the number will not change, but its scale will be significantly reduced, and only the most effective information in the feature map will be retained, thereby improving the robustness of the convolutional neural network model.

The fully connected layer is the most commonly used hidden layer of the network before the convolutional layer is proposed. Each artificial neuron in the layer establishes a connection relationship with all the neurons in the previous layer. The main feature is that there are many parameters and a large amount of calculation. In fact, it plays the role of integrating information through a large number of parameters and calculations. In a convolutional neural network, one or more fully connected layers are connected after multiple convolutional and pooling layers. Its main function is to fuse the extracted high-level features and then transform these fused features into a probability distribution. The classification result of the network is output according to the probability distribution through the output layer.

Activation functions are an important part of convolutional neural networks and are usually used in convolutional layers. The activation function is essentially a mathematical function, and its main task is to add nonlinear elements to the network model. The activation function is created by imitating the way the neurons in the human brain transmit information; that is, when the stimulation of the neuron reaches a certain threshold, the neuron will be activated to transmit the information of the neurons in the previous layer. Activation functions work in a similar way. Common activation functions are as follows:

(3) $$\begin{array}{c} \text{Sigmoid}\left(x\right)=\frac{1}{1+e^{-x}},\\ \text{Tanh}\left(x\right)=\frac{e^{x}-e^{-x}}{e^{x}+e^{-x}},\\ \text{ReLU}\left(x\right)=\max\left(0,x\right). \end{array}$$

### 3.2. Defect Detection of Agricultural Product Packaging Design with YOLOv3

The overall network structure of YOLOv3 is divided according to functions, which can be divided into backbone network and detection network. The backbone network is essentially a convolutional neural network, which is mainly responsible for the feature extraction of input images. The DarkNet-53 network is selected in the YOLOv3 model. The detection network takes the backbone network's output as an input, does multiscale prediction using regression, and outputs the full network model's detection findings.  Figure 1 shows a schematic diagram of YOLOv3's overall network topology. The backbone network DarkNet-53 is shown on the left, while the detection network on the right forecasts the outcomes based on DarkNet-53's output.

The process of performing target detection in the YOLOv3 network is as follows. The YOLOv3 network model first scales the image input to the network to a size of 416 × 416 × 3 and then inputs it into the backbone network to extract feature maps of three scales. The dimensions of the three feature maps are 13 × 13 × 1024, 26 × 26 × 512, and 52 × 52 × 256, respectively. Then, the feature maps of these three scales are input into the detection network module, the lower layer feature map performs upsampling operation, and the upper layer feature map performs feature fusion. Then, after a series of convolutional layers, three final feature maps are obtained. The dimensions of the three final feature maps are 13 × 13 × 255, 26 × 26 × 255, and 52 × 52 × 255, respectively, and these three feature maps are finally used to predict the results.

DarkNet-53 is mainly responsible for extracting feature maps of different scales. The network performs feature extraction through a series of 1 × 1 convolutions and 3 × 3 convolutions. A batch normalization layer is also included to standardize the data, speed up the network's convergence, and improve the network model's training efficiency. DarkNet-53 contains a total of 52 convolutional layers, which are composed of these 52 convolutional layers. The first is through a convolutional layer containing 32 convolutional kernels of size 3 × 3 and then through 5 sets of repeated residual block structures. Each residual block structure consists of a single convolutional layer with a set of repeatedly executed convolutional modules. Before performing the convolution operation performed separately, the zero padding operation must be completed first; that is, the zero expansion of the upper border and the left border of the input image is first performed. Then, a convolution operation with a convolution kernel size of 3 × 3 and a stride of 2 is performed. The number of specific convolution kernels is related to the depth of the network. After that, the convolution module operation is repeated, and it is repeated 1 time, 4 times, 8 times, 8 times, and 4 times, respectively. In each repeated convolution module, the convolution operation with the convolution kernel size of 1 × 1 and the number of convolutions is halved first. Then, perform a normal number of convolution operations with a kernel size of 3 × 3. This cycle is repeated for many times; that is, the feature extraction work is completed. Subsequently, a fully connected layer completes the screening of feature maps. However, the fully connected layer is actually implemented by 1 × 1 convolution; so, it can also be recorded as a convolution layer. So far, the entire network contains 53 convolutional layers, from which DarkNer-53 is named.

YOLOv3 outperforms YOLO and YOLOv2 in terms of backbone network performance. The backbone network, for starters, uses DarkNet-53 with deeper layers. DarkNet-53 employs a significant number of residual structures in addition to layer deepening. A schematic diagram of the residual structure's operation flow is given in Figure 2. The second point is that before DarkNet-53 performs the convolution operation, it will first normalize the input data of the convolution layer and then send the processed data to the convolution layer. The advantage of using this execution process is that it can greatly speed up the convergence speed of the network training.

For the detection network, we mainly rely on the feature maps of different sizes output by DarkNet-53 for result prediction. YOLOv3 uses a total of 3 feature maps for object detection. These three feature maps are located after the residual convolution module repeated 8 times by the DarkNet-53 network, after the residual convolution module repeated 8 times, and after the residual convolution module repeated 4 times. Then, use a series of convolution operations to further extract features. First, a 13 × 13 × 255 output is obtained according to the feature map with the smallest size, denoted as *y*1. A series of convolution operations and an upsampling operation are performed on the underlying feature map of DarkNet-53 to expand the size of the feature map. Then, perform a splicing operation with a feature map with a size of 26 × 26 × 512 and then go through a series of convolution operations to obtain a feature map with a size of 26 × 26 × 255, denoted as *y*2. Repeat this operation to get a new feature map, and the output size is 52 × 52 × 255, denoted as *y*3.

Finally, three different scales of *y*1, *y*2, and *y*3 are simultaneously input into the subsequent network for the final result prediction. Among them, the feature map of *y*1 is small and contains high-level feature information, which is mainly responsible for the prediction of large targets. The feature map of *y*2 is of moderate size and is mainly responsible for the prediction of medium-sized objects. The feature map of *y*3 is the largest, which contains more detailed feature information, and is mainly responsible for the prediction of small targets. It is precisely because the feature maps of different scales are used in the YOLOv3 network model that the network can achieve better detection accuracy when detecting targets of different sizes.

### 3.3. Backbone Network Improvement

The original network model of YOLOv3 was designed to conduct target detection, with the aim of detection being everyday items, which is considerably different from the target job in this topic. This subject's goal is to find flaws in the graphic design of agricultural product packaging, and the features of numerous flaws differ significantly from those of the original target object. Continuing to use the original network model, although better detection results can be achieved, it is still not optimal. In view of this, this topic will carefully study and analyze the defect characteristics and make certain improvements to the original YOLOv3 detection algorithm accordingly.

To improve the detection algorithm of YOLOv3, we first need to improve the backbone network DarkNet-53. The final output feature map size of the DarkNet-53 feature extraction network is 13 × 13, and the feature map of this scale is responsible for the detection of large objects. However, in this project, some defects have a size of more than 1000 pixels, and the detection effect of this feature map may be difficult to meet the project requirements. Therefore, this topic decided to add a residual convolution module on the basis of DarkNet-53, the internal convolution module is repeated 4 times, and the entire added module contains a total of 9 convolution operations. Aside from adding more convolutional layers, the number of repetitions of the residual convolution module of the feature extraction network must be adjusted, as well as the number of convolution kernels inside the residual convolution module. The new backbone network contains a total of 62 convolutional layers, which can be called DarkNet-62. The number of network layers is deepened, and the expressive ability of the network is enhanced.  Figure 3 is a schematic diagram of the DarkNet-62 network model.

### 3.4. Multiscale Improvement

The original network model selected 3 feature maps for the final detection result prediction. And the small-scale feature map is responsible for the detection task of large objects, and the large-scale feature map is responsible for the detection task of small objects. Due to the unsatisfactory results of previous experiments, this project plans to improve the selection of feature maps, increasing from 3 feature maps to 5 feature maps. In the previous subsection, a residual convolution module has been added, taking the output of this part as one of the selected feature maps. Then, the output of the second residual convolution module of the network model is selected as one of the feature maps, where the size of the feature map is 104 × 104. And keep the original 3 feature maps and complete the screening of the improved YOLOv3 model feature maps. A total of 5 feature maps participate in subsequent detection.

In the subsequent feature fusion process, since the 6 × 6 feature map has a size of 12 × 12 after upsampling, it does not match the 13 × 13 feature map; so, the upsampled feature map needs to be filled. Here, the method of zero padding is used to fill the upper and left sides of the 12 × 12 feature map to ensure that the subsequent feature maps can be aligned.

### 3.5. Priori Box Improvement

The YOLOv3 target detection network follows the a priori frame design of the YOLOv2 network. In the original YOLOv3 algorithm model, there are 9 a priori boxes calculated on the dataset using the *K*-means algorithm. Most of the COCO datasets are common objects and animals in life, such as TV shows, chairs, cars, cats, and dogs. YOLOv3's initial a priori frame is capable of detecting these things. The flaws in this topic are some new YOLOv3 targets, and the original a priori frame is not up to the task of detecting them.

Therefore, this project plans to reset the prior frame suitable for the agricultural product packaging graphic design defect dataset. And on the basis of the original 3, it has been increased to 5. The reason is that the different types of defects in this subject are quite different, and the sizes of other types of defects are also different. As a result, additional a priori frames are required to improve flaw detection accuracy in this subject.  Table 1 shows the distribution of the enhanced prior frame on the feature map.

### 3.6. Activation Function Adjustment

The Leaky ReLU activation function used in the original YOLOv3 network is an improved version of the ReLU activation function. But in the negative semiaxis region, Leaky ReLU presets a nonzero slope to ensure that the output of the function on the negative semiaxis is not equal to 0. This ensures that all neurons can participate in network training, and parameters can be updated in time. However, since the slope of the negative semiaxis region is preset and fixed, this makes it impossible to find the perfect parameter values that are exactly suitable for this topic, and there is no guarantee that the final result of the network is optimal.

In view of this, this project plans to use PReLU as the activation function of this defect detection network model. The advantage of PReLU is that the slope of the negative semiaxis region is a parameter that can be learned, not preset, but determined according to the data during the training of the network model. Moreover, the parameter values are fixed when the model is trained and are also constant in the subsequent testing process. The expression of PReLU is as follows:

(4) $$\begin{array}{c} \text{PReLU}\left(x\right)=\left\{\begin{array}{cc} x, & x>0\\ \frac{x}{a}, & \text{others} \end{array}.\right. \end{array}$$

## 4. Experiments

In this section, we define the dataset and detail, result of backbone network improvement, result of multiscale improvement, result of priori box improvement, and result of activation function improvement in detail.

### 4.1. Dataset and Detail

This work uses a self-made agricultural product packaging graphic design dataset. This dataset contains a total of 98,472 samples, of which 66,938 samples are training sets, and the remaining 31,534 samples are test sets. Precision and recall are used as evaluation metrics for this work. The experimental environment information is illustrated in Table 2.

### 4.2. Result of Backbone Network Improvement

As mentioned earlier, this work improves the backbone network. To verify the effectiveness of this improvement strategy (BNI), this work conducts comparative experiments to compare the defect detection performance of agricultural packaging graphic design without and with BNI improvement, respectively. The experimental results are illustrated in Figure 4.

Compared with the non-BNI improvement strategy, after using the BNI strategy, the detection network can obtain 2.1% precision and 1.5% recall improvement. This can prove the effectiveness and correctness of this work using the BNI improvement strategy.

### 4.3. Result of Multiscale Improvement

As mentioned earlier, this work improves the multiscale prediction. To verify the effectiveness of this improvement strategy (MSI), this work conducts comparative experiments to compare the defect detection performance of agricultural packaging graphic design without and with MSI improvement, respectively. The experimental results are illustrated in Figure 5.

Compared with the non-MSI improvement strategy, after using the MSI strategy, the detection network can obtain 1.5% precision and 1.1% recall improvement. This can prove the effectiveness and correctness of this work using the MSI improvement strategy.

### 4.4. Result of Priori Box Improvement

As previously stated, this effort enhances the priori box. This work performs comparison experiments to compare the defect detection performance of agricultural package graphic design without and with PBI improvement, respectively, to validate the usefulness of this improvement approach (PBI). The experimental results are illustrated in Figure 6.

Compared with the non-PBI improvement strategy, after using the PBI strategy, the detection network can obtain 1.7% precision and 1.3% recall improvement. This can prove the effectiveness and correctness of this work using the PBI improvement strategy.

### 4.5. Result of Activation Function Improvement

As mentioned earlier, this work improves the activation function. To verify the effectiveness of this improvement strategy (AFI), this work conducts comparative experiments to compare the defect detection performance of agricultural packaging graphic design without and with AFI improvement, respectively. The experimental results are illustrated in Figure 7.

Compared with the non-AFI improvement strategy, after using the AFI strategy, the detection network can obtain 1.0% precision and 0.8% recall improvement. This can prove the effectiveness and correctness of this work using the AFI improvement strategy.

## 5. Conclusion

Computer graphics and image processing technology are maturing in tandem with the rapid advancement of information technology. In graphic design, the use of computer graphics and image processing technology can help to simplify the process, enhance the design effect, and better the design expression. People's expectations for graphic design quality are rising in tandem with the manufacturing industry's rapid growth; although, flaws are unavoidable in the design process. Graphic design defects not only affect the appearance itself but also affect the use; so, enterprises pay special attention to product quality inspection to ensure the quality of products. At the same time, the quality inspection results are analyzed to further improve the graphic design process and reduce the occurrence of defects. As a result, this study examines the use of a convolutional neural network as a computer graphics and image processing technology in defect identification in graphic design, as well as the current position. To complete the enhancement of the YOLOv3 network model, this work uses the packaging design of agricultural products as an example. The network model is presented to improve the direction of this topic based on the experimental findings of the original YOLOv3 and an in-depth analysis of the characteristics of various agricultural product packaging graphic design faults. It includes the improvement of the backbone network, the improvement of the feature map, the improvement of the prior frame, and the improvement of the activation function. Finally, the validity and feasibility of the model improvement are proved by experiments.

## Figures and Tables

**Figure 1:** The structure of YOLOv3.

**Figure 2:** The structure of residual module.

**Figure 3:** The structure of DarkNet-62.

**Figure 4:** Result of backbone network improvement.

**Figure 5:** Result of multiscale improvement.

**Figure 6:** Result of priori box improvement.

**Figure 7:** Result of activation function improvement.

**Table 1:** Improved prior box.

Priori box	Feature map size
352 × 1127, 465 × 272, 725 × 787	6 × 6
189 × 797, 228 × 195, 296 × 62	13 × 13
104 × 42, 122 × 103, 147 × 132	26 × 26
57 × 172, 76 × 77, 87 × 427	52 × 52
27 × 26, 42 × 40, 52 × 62	104 × 104

**Table 2:** Experimental environment information.

Name	Parameter
CPU	Intel i9-9900K
GPU	GeForce RTX 2080Ti(11GB)
Memory	32GB
Framework	PyTorch 1.6

## Data Availability

The datasets used during the current study are available from the corresponding author on reasonable request.
